The article "Determinants of Unverified News Sharing on Social Media and Its Effects on Corporate Image" was published in 2022. Journal: Front Psychol.

# Determinants of Unverified News Sharing on Social Media and Its Effects on Corporate Image

**DOI:** 10.3389/fpsyg.2022.937104

**Published:** 2022-07-15

**Authors:** Zhe Zhang, Shamim Akhter, Mohammed Ali Al-Abyadh, Phan The Cong

**Affiliations:** ^1^School of Humanities and Law, North China University of Technology, Beijing, China; ^2^Renmin University of China, Beijing, China; ^3^School of Languages, Civilisation and Philosophy, Universiti Utara Malaysia, Sinkot, Malaysia; ^4^College of Education, Prince Sattam bin Abdulaziz University, Alkharj, Saudi Arabia; ^5^College of Education, Thamar University, Thamarj, Yemen; ^6^Department of Economics, Thuongmai University, Hanoi, Vietnam

**Keywords:** social consciousness, entertainment, unverified news sharing, corporate image, workplace stress, CSR

## Abstract

Social media channels are interactive channels that let users spread content, participate, and generate positive or negative news. In this era of social media (SM), organizations run structured and systematic campaigns to shape their corporate images. The present study examines the role of social consciousness (SC) of employees, entertainment (Ent), and altruism (Alt) on unverified news sharing (UVN) with the mediation of corporate image (CI) and the moderation of workplace stress (WS). We conducted the study on 375 employees of the social media teams in the corporate sector in China. The sampling technique used in this study is convenience sampling. We carried out data analysis using structural equation modeling (SEM) with the help of Smart PLS (Partial Least Square) software. The results reveal that the entertainment and altruism of employees affect UVN. However, the direct negative effect of social consciousness of employees and CI on UVN came out to be insignificant. The findings also show that CI mediates the relationship between the social consciousness (SC) of employees and UVN, altruism and UVN, and entertainment and UVN. The moderating role of WS between CI and UVN is significant. Theoretically, the study contributes to the literature by examining the effect of different determinants of UVN on SM on the role of CI and WS. Practically, the present study provides implications for the managers and the organizations. The study finds that Alt is an essential factor that fosters UVN and CI; therefore, altruistic values of the employees should be instigated to reduce the flow of UVN.

## Introduction

“Managing stakeholder responsibility for acceptable and negligent activities associated with environmental, moral, and societal issues in a way that provides business benefit” is what Corporate Social Responsibility (CSR) entails (Huo et al., 2022). Therefore, it is associated with all the good things an organization should do and refrain from what is not suitable for the organization. These should align with society’s expectations and provide a competitive edge to the organization. There should be an approach for avoiding the wrong things for the organization and getting excellent results in the long run (Huo et al., 2022). CSR is important as many organizations deploy it to fulfill the stakeholders’ demanding needs. Corporate Image (CI) is one of those CSR practices that shape the organization’s image and reputation. Therefore, it has been studied in various contexts so far. In times of digitalization, SM has been a popular source of news dissemination. The management of corporate organizations is now focusing on such SM platforms to devise and predict socially responsible management practices that may regulate SM use. It is also understood that SM gives news a thrust of spread about any organization instantly. It becomes the responsibility of the management to monitor the factual news and filter out the unverified or fake news, which harms the CI of the organizations (Garcia-De los Salmones et al., 2021).

Foremost of all, it is necessary to understand what unverified news is shared on SM. It also determines the factors that amplify or reduce UVN on SM. It is also necessary to determine which factors aid in spreading or stopping UVN. Therefore, we designed this study. SM allows for two-way contact and a discussion between companies and stakeholders. It represents a new type of connection (Abitbol and Lee, 2017). Millions of stakeholders, including businesses and individuals, interact daily in this digital environment, resulting in exceptional communication. As people are directly involved in communication, the conventional difference between corporations and third party-controlled media becomes blurred. Therefore, it becomes challenging to control the news-sharing behavior of the users. People equally share verified and unverified news on social networking sites and start believing in such information due to their uncontrolled spread. Unverified news sharing (UVN) is now becoming a global problem. Even if this behavior is not new, it has become more concerning due to the widespread use of SM, which allows for interaction and the spread of new beliefs. In this era, people on SM may promote views or propagate news by sharing, liking, or retweeting.

Unmanageable information constantly subjected people to news, by independent authors. Therefore, SM has become a vehicle for quickly disseminating false information and unverified news (Rampersad et al., 2019). Lazer et al. (2018) demonstrated that SM is a powerful tool for disseminating large amounts of unfiltered content, facilitating the spread of false information, and opening up the possibility of altering the populace’s understanding of reality through the propagation of unverified news content. According to Duffy et al. (2020), Unverified fake news is made-up content that mimics actual news and is presented delicately to fool the public into assuming it is true.

In today’s internet environment, UVN has spread like wildfire. It shows that even certain government officials and people disseminate such material to a large audience to achieve their agenda (Wasserman and Madrid-Morales, 2019). UVN has impacted almost every part of our lives. Since news passes considerably faster and further than before web-based technology, the ubiquity of SM magnifies this tendency (Apuke and Omar, 2021). SM provides users the incredible comfort of sharing news with just a click, frequently without scrutinizing the material. Individual conduct, such as distributing news before verifying it, is a significant contributor to the spread of disinformation. Understanding people’s UVN on social networks is critical in combating the disturbance caused by the people. Several additional concepts like disseminating wrong information and fake news were used alternatively in previous studies to UVN. Disparities between them must be understood. UVN stresses that people exchange information without validating it, which could be inaccurate or misleading (Huang et al., 2022). Persons’ sharing of false news that is made without the aim of causing harm is referred to as misinformation sharing. At the same time, sharing fake news was crafted to engage the readers misleadingly (Huang et al., 2022).

Ordinary people find it increasingly difficult to distinguish between unconfirmed news, false news, and facts. Due to the quick expansion of SM platforms and news overload, it happens. When people discover their knowledge is erroneous, they rarely spread disinformation or fake news on purpose. Nonetheless, it is relatively normal not to know the truth of information and to share it without verifying it (Laato et al., 2020). What factors lead the people to share unverified news, especially in the organizations? On the side, it also raises concerns for the socially responsible organizations what extent these determinants of UVN impact the CI of these organizations. Previously, a few scholars looked into the determinants of news sharing on SM (Thompson et al., 2020), which supported the current context of organizational management of employees influencing CI. As suggested by Thompson et al. (2020), certain factors determine the behaviors associated with news sharing. Among these, the social consciousness (SC) of employees is given prime importance. Therefore, the authors tried to scale down its impact on UVN behavior. Employee SC describes how enterprises appreciate social value, strive to establish relationships with various stakeholders, and evaluate performance on social affluence and organizational success.

Therefore, socially conscious organizations and their employees seek opportunities to forecast and solve social problems by aligning their interests with the different social players involved (Pandey and Gupta, 2008). With this alignment, the authors draw a relationship between the SC of employees with UVN behavior in current research. This relationship is developed by keeping in mind the significance of SC, which may inhibit such behavior of sharing unverified news. Along with this type of consciousness, this study also tries to scale down the impact of other attributes of using SM on UVN, such as entertainment (Ent) and Alt.

Users of SM sites like Facebook reported being motivated by various factors, including a want for Ent, a desire to be informed, and learning about their friends’ social activities (Islam et al., 2020). Along with the Ent aspect, Alt is also an attribute of sharing unverified news on SM (Islam et al., 2020; Huang et al., 2022). Most of the previous study on unverified news have taken a psychological approach. The first experimental path used the theory of uses and gratification to see UVN as behavior driven by various needs, including sociability, self-promotion, spending leisure time, Ent, and Alt (Balakrishnan et al., 2021). The term altruism (Alt) states the behavior of giving anything to anyone in return for nothing, whether it be a favor or any incentive (Plume and Slade, 2018). This kind of behavior is prevalent in society because people think about themselves as a torchbearer of humility and, in return, need no reward. In news sharing, this kind of behavior entails giving information or the news on SM without thinking about obtaining a reward from the connected people on SM. They may share news on SM platforms from humility and helping others, but they share unverified news (Apuke and Omar, 2021). It leads to sharing such news, which is fake and wrong, while it may harm the people getting that news.

Sometimes shared news due to Alt may be beneficial, but most of the time, it ends in chaos. The behaviors of employees influence organizational success, which may lead to actions that are not in line with the objectives of the organization’s CSR. For the sake of the social responsibility of the organizations, CI is one of the leading indicators which leads to socially responsible management of organizations (Kim et al., 2020). The CI of the firms is related to the interactions of behaviors, beliefs, feelings, and knowledge of the employees of the firms. It helps provide several benefits to the organizations, and it can also help the organization do well even in times of crisis. Therefore, the news-sharing behaviors of the employees, such as SC, Ent, and Alt, influence it (Bataineh, 2015). After establishing the possible link between SC, Ent, Alt, and UVN, it is necessary to determine the mediating factors that may enhance or inhibit UVN on SM. Garcia-De los Salmones et al. (2021) suggested a considerable gap in previous research and investigations about the interconnectedness of these factors involved in UVN. Therefore, to fill this gap, this study tries to find out the positive and negative effects of SC, Alt, and Ent of UVN behaviors. In this wake study, this research also tries to find out the mediating impact of CI on the behavior of UVN. This research comprehensively addresses the concerns about behaviors of employees which lead to such sharing of unverified news on SM.

## Theoretical Underpinning

We developed the current model of the study from the perspective of Uses and Gratification Theory (UGT) which was proposed by the researchers (Blumler et al., 1974). According to the theory, it becomes necessary first to understand why people utilize various media platforms. The idea of UGT addresses the question of the defining aims due to which people select different media to achieve their goals. The theory helps in figuring out how to use that media. It also affects the motivations of the people who use the media because they are using it (Halpern et al., 2019). UGT helps explore a person’s needs with which they try to connect with other people. It also influences the selection sense of people to use the media of their own choice, providing the assessment of the information gained or disseminated through that specific media (Rubin et al., 2019).

The UGT was first originated and designed for the conventional media available. However, currently, it also provides the basis for the research on online mediums and SM with the help of the internet. The researchers involved in SM studies get theoretical support from UGT to resonate with the benefits that individuals and groups can gain from levels from using SM sites (Thompson et al., 2020). Introne et al. (2018) identified knowledge-seeking, earning, amusement, and social interaction as benefits of using SM. Similarly, few researchers discovered the link of SM networking to knowledge probing, relationship maintenance, and peer approbation (Dunne et al., 2010). Some scholars identified Ent, SC, information-seeking behavior, Alt, and socialization as some uses of SM and its usage through different platforms (Thompson et al., 2020).

According to a study by Apuke and Omar (2021), news-sharing behavior has a link to SC and Alt gratification. Conversely, persons with more motivation for enjoyment, socialization, and SC spread the news on SM more frequently. Previously, some researchers tried to evaluate news-sharing behavior with socialization and interpersonal communication, which hinted at a positive relationship (Chiu et al., 2006). Authors argue that specific approaches to using SM influence sharing of unverified news. These approaches are assumed to be happening due to SM. High engagement of social users leads to sharing content that is not verified before. This synchronization assumption is based on the previous research based on UGT. The beginnings of U&G theory may be dated directly to mass communication research in the 1950s and 1960s when the field shifted attention from primarily focusing on the effects of media on its audiences to how viewers play any part in media selection (Ruggiero, 2000). Therefore, audience members were more active than passive in their media consumption. Schramm (1965) argued that children’s television viewing habits differed significantly based on their circumstances, such as overall cognitive talents and connection with their parents. People are most often left despondent and distanced due to our modern society’s expectations, according to Katz and Foulkes (1962). Consequently, people turn to mass media to fill specific psychological and social requirements that may miss (Katz and Foulkes, 1962). Other people go to the movies to relax over their difficulties or forget, showing using the medium to escape reality. Katz et al. (1973) established the UGT to comprehend better the complex reasons people use certain media. The UGT’s main aim is to describe how and why people intentionally pick some types of media over others to meet their needs (Katz et al., 1973). Social media (SM) arose because of advancements in Internet technology. According to Nov et al. (2010), the capacity to empower individuals to generate their material is one of the most appealing aspects of SM. The other most valuable aspect of SM usage is turning the audience from a passive to an active state of participation (Nov et al., 2010). It inspired researchers and other related work to look at UGT through the lens of SM.

As a result, socialization, SC, informativeness, enjoyment, Alt, sharing of information, and status-seeking are the most common UGT variables discovered in SM studies (Islam et al., 2020). We used some of these gratifications in our work. Consequently, the current study develops a thorough predictive model that reveals a link between Alt, enjoyment, SC, and the dissemination of unconfirmed news. This research also supports the theory of reasoned actions (TRA), as suggested by Mustățea and Balaban (2019). UGT provided the basis for the likely reasons for sharing unverified news on SM. This theory provides the basis for SC, Alt, and Ent, due to which employees share unverified news on SM.

### The Social Consciousness of Employees and Unverified News Sharing

The consciousness of employees is attributed to the social and environmental contexts. For their differentiation, SC is a person’s care for his or her society and its members (Ladhari and Tchetgna, 2017), while environmental consciousness refers to a set of psychological characteristics that influence a person’s intentions to take part in pro-environmental activities and make sustainable consumer choices (Martínez García de Leaniz et al., 2018). Socially conscious people understand the influence of others on themselves and their influence on others. Their awareness, compassion, and understanding of other people’s well-being distinguish them. Moreover, it includes their improvements in the community, quality of life and economic advancement, and environmental protection (Garcia-De los Salmones et al., 2021).

Such people operate accordingly with their interests and social concerns, with the ecology playing a significant role. As a result, while environmental and social values are distinct concepts, they are intertwined. Individuals who respect communal or pro-social characteristics are more worried about the environment and have more excellent pro-environmental sentiments (Garcia-De los Salmones et al., 2021). Consciousness might affect perceptions of SM networking, and in this case, SM sharing. According to some scholars, understanding and alteration in their point of view resulted in varying levels of the SC, ranging from passive citizens to individuals who have a deep sense of connectedness with each other (Martínez García de Leaniz et al., 2018). Whenever an individual knows that his/her activities in the social environment influence others, they get motivated to act accordingly. They either act individually (engrossed level) or collaboratively (collaborative levels). It includes telling experiences, perceptions, and thoughts and having taken part in a field of shared experience with social communities. Varying levels of awareness evolve in response to what the social situation may represent, and consciousness grows as personal experiences are shared publicly. Because SM is public media and allows individuals to discuss ideas and interests and form communities, it can help accelerate this happening change through the active involvement of the people based on these concerns (Kim et al., 2019).

Earlier studies reported that people on SM became more sensitive to ethical and environmental concerns and that sustainability reports encourage consumer participation. Therefore, as a result, the more socially conscious employees are, the more likely they are to engage with CSR content on social accounts (Uzunoğlu et al., 2017). These points can apply to the setting of our study. Individuals with higher levels of consciousness, both at the environmental and social levels, are more likely to seek knowledge about valuable goods and act as a source of disseminating such news (Aldwairi and Alwahedi, 2018). Because of the options for engagement, dialogue, and shared space provided by various media, such people would be inclined more to take part in sharing news on the SM, whether verified, resulting in increased levels of consciousness. Therefore, we developed the following hypothesis to explore the association between both.

*H1*: Social consciousness of employees has a negative impact on unverified news sharing.

### Entertainment and Unverified News Sharing

Using SM is a system of information sharing pleasantly, so it is influenced, at least to some extent, by characteristics like delight, pleasure, and Ent (Mäntymäki and Islam, 2016). A user’s desire for amusement or Ent is fulfilled, for example, by sharing humorous stories with their friends to make fun of politicians and celebrities (Rieger and Klimmt, 2019). The individuals who have an urge to enlighten and assist the other individuals are worried about the accuracy and dependability of the news they tend to provide. The individuals who like to have fun might not even feel the same way (Islam et al., 2020). We characterize SM platforms as a multifunctional arena, implying that they could be used for Ent, sharing, and reading news. The sense is developed based on the affirmance lens (Norman, 1988). The people who use SM to kill time affording, take part in an activity that interests them, and get away from their daily routines, enjoy themselves. The benefit of using SM is entertaining and relieving mental tension and stress. According to the latest study, individuals use SM for Ent, relaxation, and amusement when sharing (Baek et al., 2011). A study conducted by a small group of academics discovered a correlation between the age of SM and Ent. According to the same research, people used the like button feature on Facebook to express their thoughts on many topics (Kim et al., 2015). Previously, Talwar et al. (2019) identified that both are not connected aspects like they do not influence each other, or it can also be extracted that there was no sense of Ent in sharing unverified news on SM by the users.

Nonetheless, it was also clear from some of the researchers’ work analysis that there was an element of enjoyment and Ent in the information dissemination socially interactively. These results showed that people on SM have an urge to use it to kill their spare time and for Ent (Talwar et al., 2019). Islam et al. (2020) also assessed that users of SM websites use it as an entertaining activity that allows them to locate valuable information that they then share with others on SM. During pandemics, a desire to have Ent motivated a significant quantity of information transmission, including SM interactions. Comedy as a buffering technique often fuels it in harsh circumstances or keeps up with current material (Chiodo et al., 2020).

A survey of pandemic-related Twitter messages discovered that the users of the Twitter platform tweeted funny content regarding the pandemic during the current pandemic, and the proportion of such tweets was about 6.1% in a lighter mode (Kouzy et al., 2020). While amusement is a positive thing, pursuing Ent as a goal is unconcerned with the accuracy of the news presented if the content is amusing. As a result, it is reasonable to assume that using SM for Ent contributes to more unverified material being shared (Islam et al., 2020). Although, there has been no research found previously which evaluated the direct association of Ent as a predictor of UVN on SM. Therefore, the authors tried to find out the association between them both. So, the study developed the following hypothesis.

*H2*: Entertainment has a positive association with unverified news sharing.

### Altruism and Unverified News Sharing

Altruism is the act of giving anything to someone without expecting something in return. Alt could be defined as the act of providing news and information without expecting anything in return. In motivational experiments examining information and knowledge sharing in SM, Alt is among the most commonly investigated elements (Martínez García de Leaniz et al., 2018). Alt is the most significant incentive about which individuals actively seek knowledge and provide responses to the others, according to Ma and Chan (2014). According to previous research, users who share news are driven by the psychological resonance the news has on them, its significance for the receiver, and the user’s purpose in offering counsel or caution (Apuke and Omar, 2020). Such impulses are distinctive to individuals who are frequently labeled as having a high level of Alt. People tend to help one another, which is visible when sharing information, regardless of if it is genuine, as long as it offers preventive steps, in particular situations (Apuke and Omar, 2020). Alt is a motive that shows an individual’s desire to help others, as opposed to concern for customers, in that those driven by Alt offer news just for the pleasure of helping others. The altruistic incentive has been explored and defined through the research on SM platforms to disseminate information (Alhabash et al., 2012). According to the existing literature, there is also an altruistic reason for sharing within the SM ecosystem (Wu and Pearce, 2016).

When people share expecting nothing in return, they act altruistically. Alt is the act of disseminating news and information while asking nothing in return. The altruistic person constantly considers how they might assist others (Plume and Slade, 2018). It shows that if someone is looking for information or news, an altruistic person is always eager to share it without asking for anything. Altruistic conduct has been carefully examined and recorded in a study on knowledge, information, and news sharing. For example, studies revealed that Alt is directly associated with volunteering information collecting and dissemination, meaning that SM users will contribute and expect nothing in return (Ma and Chan, 2014). Research supports this viewpoint that disseminating news on social networking platforms correlates with organizational cohesiveness. The emotional effect and significance of the news on the recipients [Duffy et al. (2020) also motivated individuals who engage in these behaviors]. According to a recent study, individuals tend to disseminate information to improve others without considering whether it is genuine, as long as it includes certain precautionary actions based on specific themes (Apuke and Omar, 2020). Resultantly, a link involving Alt and spreading unverified news might be expected. We have hypothesized that persons with a more altruistic perspective are more prone to broadcast Unsubstantiated material on SM while striving to help others (Apuke and Omar, 2021). A hypothesis was built and given below.

*H3*: Altruism has a positive association with unverified news sharing.

### Corporate Image

When unfavorable information is linked to a corporation, the CI can influence UVN intentions. Study showed that a positive CI was identified as a resource that results from the interconnectedness of the feelings, knowledge, beliefs, and conceptions of the individuals associated with the organization. It could provide the organization with an advantage of a valuable asset during critical times. Consumers develop opinions and inferences of responsibility for faulty or hazardous products on their own, and these beliefs and attributions serve as the foundation for brand assessments and behavior (Thompson et al., 2020). Customers rely on the information, such as business relationships and previous CI. It also helps develop an impact on customers’ minds about the organizations (Insch and Black, 2018). Suppose a stakeholder has a positive effect on the company? In that case, he or she may give it the ‘benefit of a doubt,’ assigning it less blame for a crisis than a company with an unknown or unfavorable image; this should lead to minor damage to the organization’s reputation (Thompson et al., 2020). Rhee and Haunschild (2006) take a different approach, speculating that enterprises with a strong reputation may face a more excellent price in certain situations. They discovered that a high-quality company reputation has a detrimental effect on market responses to production problems in the business. As a result, a high reputation does not always protect businesses from market variances. The research only looked at measuring reputation quality.

As the authors acknowledge, it can be a study’s drawback because many other factors influence an organization’s reputation. CI is among the most significant strategic assets available to businesses. It provides fertile ground for establishing a long and robust competitive edge over competing brands. Bataineh (2015) found that its CI aids customers’ understanding of a company’s quality, which reduces indecision during the purchasing decision. Plume and Slade (2018) studied that CI negatively influences the intention to share fake news and could also mediate the relationships between determinants of news sharing and intention to share the news (Plume and Slade, 2018). Therefore, the following hypotheses were developed.

*H4*: Corporate image harms unverified news sharing.

*H5*: Corporate image mediates the relationship between the social consciousness of employees and unverified news sharing.

*H6*: Corporate image mediates the relationship between entertainment and unverified news sharing.

*H7*: Corporate image mediates the relationship between altruism and unverified news sharing.

### Workplace Stress

There are two types of workplace stressors: physical and psychosocial. Pollution, poor lighting, a lousy workplace or work arrangement, and ergonomic problems, including suboptimal body posture, are all physical stresses. Psychological stresses are, without a doubt, the most common stressors. Excessive workplace expectations, rigid work hours, poor job control, bad work size and layout, harassment, bullying, and job insecurity are just a few examples. WS affects the employee, but also harms the company’s performance. Employees’ health, emotional health, and behavior are all affected by WS. These affects happen in stages, starting with discomfort in reaction to stresses. Stress causes high blood pressure and psychological issues, which raises the risk of cardiovascular disease, substance misuse, and mental illnesses (Birhanu et al., 2018). WS also has a consequence on the health of employees who suffer from coronary heart disease, anxiety, or cancers. Because of WS, companies will suffer damage due to employees’ unhappiness, pessimism, higher turnover, and unavailability. Prior studies have looked at the link between WS and burnout in nurses, bank managers, and doctors. Other research has discovered that WS impacts job satisfaction and the employees’ sleep quality (Xie et al., 2021). WS harms individuals’ mental, behavioral, and physical health. It harms motivation, confidence, and effectiveness.

Furthermore, it has a detrimental association with satisfaction, which reduces one’s motivation to work and leads to poor effectiveness. Workers who are stressed are more likely to have poor health and have negative job experiences. As a result, they have less energy to concentrate on their work, and their performance suffers. The detrimental effects of work stress may jeopardize employees’ health on their psychological and physical states, including harmed mental functions, quick memory loss, and, in difficult situations, impeded recollection of knowledge and disturbed concentration (Hayajneh et al., 2021). WS has been proved to be a regulating factor of employees’ performance, and it could also deteriorate the CI. Therefore, in the current study, it could have a moderating effect on the employees’ UVN behavior, damaging the CI. So, the following hypothesis was developed.

*H8*: Workplace stress negatively moderates the relationship between corporate image and unverified news sharing.

A conceptual framework of this research is devised and given in Figure 1.

**Figure 1:** Theoretical framework.

## Methodology

This section specifies the methods undertaken to examine the impact of the SC of employees, Ent, and Alt on UVN. We examined the previous relationships in mediating and moderating corporate image and WS mechanisms. After analyzing the underlying study objectives, the researcher adopted a deductive approach and a quantitative design to mitigate any biases and ensure the credibility and reliability of the data. A survey technique was used for data collection from the study participants. The survey form was assessed for precision and clarity to ensure data rationality (Hair et al., 2017). We circulated a total of 500 survey forms to the participants. The study was conducted on the corporate sector employees working at various corporations across China. In particular, the population targeted for the present study was the employees of the media cells of different organizations handling the SM campaigns for their respective organizations. This sector is considered the population because, these days, most organizations maintain their online and SM marketing through Facebook ads, Instagram accounts, etc. (Dian et al., 2021; Li et al., 2021; Mason et al., 2021a,b). A non-probability convenience sampling strategy was used to devise the sample size. This strategy was used because it helps the researcher gain data within a shorter period and in a less costly way (Scholtz and Scholtz, 2021). Moreover, the unit of analysis of this study was individual, and the time horizon was cross-sectional, so the data were got at one point only (Hair et al., 2014).

We collected the data through self-administered surveys. For this purpose, we approached the corporate firms having SM marketing cells for their advertisement on the internet. The researchers approached the organizations with prior appointments from the administration. With their acceptance, the SM marketing department employees were contacted. We informed them about the purpose of the study and took their consent to being part of it. Those who agreed were distributed the forms. The potential respondents were explained the questions. They were ensured about the anonymity of their responses and that the survey will only be used for the research purpose. The social desirability bias was tried to minimize by telling the respondents that questions in the survey have no right or wrong answers. The data collection process took 3 to 4 weeks to complete. Out of the 500 survey forms that were initially circulated, 375 were properly filled and were considered for analysis. One hundred twenty-five forms were discarded. The overall response rate was 75%. Data from these survey forms were then arranged and assessed with the help of specialized statistical software. We tested the proposed hypotheses through the Smart PLS 3.3.3 software. Using this software, an SEM technique was used to confirm the presence/absence of relationships between the constructs of the study. Reason behind using this software was that it significantly helps the researcher formulate a path model, which aids in evaluating the data effectively (Cho et al., 2020). The path model comprises the measurement and structural models. The measurement model evaluates data reliability, whereas the structural model examines the validity of the hypotheses using *p* values and t-statistic values.

### Measurement

We adopted the measurement instruments from studies conducted within a similar context. A Likert scale comprising 5 points was used to measure the variables. The scale of social consciousness (SC) had three items (“I consider myself a person concerned about what happens in society,” “I consider myself a person committed to my society,” and “I consider myself to be a socially conscious person”), and it was adopted from Garcia-De los Salmones et al. (2021). There were three items on the Entertainment (Ent) scale, and it was adopted from Islam et al. (2020). Items included in this scale were “I share an information or news on SM when the news is entertaining,” “I share information or news on SM when the news is catchy and resonates with me,” and “When I see exciting news, I share it on SM.” Altruism had 6 items, and its scale was adopted (Büssing et al., 2013). Items included “I help others even when there is no direct benefit to me,” “When I see suffering, I try to find ways to alleviate it,” “When I see individuals in need, I think about how to relieve their distress or meet their needs,” “If someone I do not know intends to borrow something really important to me, I will lend it to them nonetheless,” “I can relinquish my material goods in favor of the common good,” and “When I see individuals in need, I ask them how I can help.” There were four items on the scale of Unverified News Sharing (“The pace of work at my workplace is high,” “I have difficulties not thinking of my work in my free time,” “I feel high demands of performance in my work,” “I can myself decide when and where to carry out my tasks,” “I often feel stressed at my workplace,” and “Do you feel that you are bullied at your workplace”). It was adopted from Islam et al. (2020). Items included: “I often share information or news without checking its authenticity,” “I share information or news without checking facts through trusted sources,” “I share information or news without verifying that it is true,” and “I share information or news even if sometimes I feel the information may not be correct.” The CI had three items (“I have a good image of the company,” “I value the company positively,” and “My attitude towards the company is favorable”), and its scale was adopted from Garcia-De los Salmones et al. (2021). Whereas the scale of WS comprised 6 items, and it was adopted from Lagrosen and Lagrosen (2022).

### Demographic Profile

Table 1 demonstrates the demographic characteristics of the respondents. It can be viewed that there were 213 males and 162 females who agreed to be a part of this study. The participation of males was 56.80%, and the female participation ratio was 43.20%. The age distribution shows that 84 individuals were between 20 to 30 years of age. Individuals numbered 161 belonged to the age group of 31 to 40 years. Seventy-five individuals were aged between 41 and 50 years, and 55 were above 50. 68 participants had a bachelor’s education, 199 had a master’s degree, whereas 108 had a Ph.D. or some other qualification. Besides this, 86 individuals had an organizational tenure of less than one year, 125 individuals had a tenure of 1 to 3 years, 118 had a tenure of 4 to 6 years, whereas employees with an organizational tenure of over six years were 46.

**Table 1:** Demographics analysis.

**Demographics**	**Frequency**	**Percentage**
**Gender**		
Male	213	56.80%
Female	162	43.20%
**Age (years)**		
20–30	84	22.40%
31–40	161	42.93%
41–50	75	20.00%
Above 50	55	14.67%
**Education**		
Bachelors	68	18.13%
Masters	199	53.07%
Ph.D. and others	108	28.80%
**Organizational Tenure (years)**		
Less than 1	86	22.93%
1–3	125	33.33%
4–6	118	31.47%
Over 6	46	12.27%

*N = 375 s.*

## Data Analysis and Results

### Measurement Model

The output of the measurement model in the presence and absence of the moderator can be viewed in Figures 2, 3, respectively. The figures provide a visual demonstration of the relationships between the constructs of this study.

**Figure 2:** Output of measurement model without moderation. SC, Social Consciousness of Employees; Ent, Entertainment; Alt, Altruism; UVN, Unverified News Sharing; and CI, Corporate Image.

**Figure 3:** Output of measurement model with moderation. SC, Social Consciousness of Employees; Ent, Entertainment; Alt, Altruism; UVN, Unverified News Sharing; CI, Corporate Image; and WPS, Workplace Stress.

Table 2 provides a thorough assessment of the direct model. It comprises the values of factor loadings, VIF, AVE, composite reliability, and Cronbach’s Alpha. It can be viewed that all factor loadings ranged between 0.738 and 0.915, which is well above the minimum threshold value of 0.70 suggested by Bollen (2019). Moreover, Hair et al. (2017) suggested that the desirable values of VIF must be less than 5. It can be viewed that all VIF values were below 5. Based on these observations, it can be found out that the data had no collinearity issues. The Cronbach’s Alpha and composite reliability indicators were used to confirm data reliability. Taber (2018) posited that the desirable values of Cronbach’s Alpha must be greater than 0.70. All alpha values successfully met this assumption. As far as composite reliability is concerned, Peterson and Kim (2013) stated that all composite reliability values must be greater than 0.70. The results from the table show that all values of composite reliability were above 0.70.

**Table 2:** Model assessment (direct model).

	**Factor loadings**		**VIF**	**Construct reliability and validity**		
				***α***	**Composite reliability**	**AVE**
**Social consciousness of employees**	SC1	0.860	2.086			
	SC2	0.870	1.893	0.847	0.907	0.765
	SC3	0.894	2.239			
	Ent1	0.892	2.283			
**Entertainment**	Ent2	0.889	2.315	0.871	0.921	0.795
	Ent3	0.894	2.322			
	Alt1	0.910	4.239			
	Alt2	0.859	2.940			
**Altruism**	Alt3	0.890	3.858	0.925	0.943	0.736
	Alt4	0.910	4.034			
	Alt5	0.891	3.692			
	Alt6	0.759	1.510			
	UVN1	0.854	1.984			
**Unverified news sharing**	UVN2	0.915	3.226	0.870	0.911	0.719
	UVN3	0.809	1.952			
	UVN4	0.808	2.110			
	CI1	0.738	1.339			
**Corporate image**	CI2	0.854	1.696	0.736	0.850	0.655
	CI3	0.832	1.526			

*SC, Social Consciousness of Employees; Ent, Entertainment; Alt, Altruism; UVN, Unverified News Sharing; CI, Corporate Image; VIF, Variance Inflation Factor; α, Cronbach Alpha; and AVE, Average Variance Extracted*.

Moreover, the researcher used average variance extracted (AVE) to assess the presence of convergent validity. Shrestha (2021) suggested that all AVE values must be above 0.50. The results show that all AVE values were well above the specified threshold limit. Hence, indicating convergent validity.

Table 3 shows the tests that were undertaken to confirm the presence of discriminant validity. For this purpose, the HTMT ratio and the Fornell and Larcker criterion were used. The desirable value of HTMT must be less than 0.90 (Franke and Sarstedt, 2019). It can be viewed that all values of HTMT lay within the range of 0.428 and 0.882. As far as the Fornell–Larcker test is concerned, a general rule is that the values at the top of each column must be higher than the ones below them (Fornell and Larcker, 1981). This assumption was satisfied, and therefore, it was established that discriminant validity was also present in the data.

**Table 3:** Discriminant validity.

**Fornell–Larcker criterion**						**Heterotrait–Monotrait ratio**					
Constructs	**Alt**	**CI**	**Ent**	**SC**	**UVN**	**Constructs**	**Alt**	**CI**	**Ent**	**SC**	**UVN**
**Alt**	0.858					**Alt**					
**CI**	0.533	0.810				**CI**	0.635				
**Ent**	0.586	0.506	0.892			**Ent**	0.654	0.623			
**SC**	0.433	0.771	0.371	0.875		**SC**	0.488	0.982	0.428		
**UVN**	0.583	0.695	0.588	0.515	0.848	**UVN**	0.632	0.834	0.662	0.578	

*N = 375, SC, Social Consciousness of Employees, Ent, Entertainment, Alt, Altruism, UVN, Unverified News Sharing, and CI, Corporate Image.*

We assessed the sustainability of the model and its predictive relevance by observing the r-square and q-square values. Hair et al. (2014) indicated that an r-square value close to 0.50 suggests high model sustainability. The R-square values of the outcome variables, i.e., CI and UVN, were 0.661 and 0.577. It shows that the model sustainability was high. On the other hand, to ensure significant predictive relevance, the q-square values must be higher than 0. It was observed that both the dependent variables, i.e., CI and UVN, had q-values of 0.412 and 0.389, respectively. Furthermore, the inner VIF values were also examined. To eliminate collinearity, the inner VIF values must be less than 5 (Legate et al., 2021). All inner VIF satisfied this assumption. Thus, it was established that there were no collinearity issues in the data.

### Structural Model

Figures 4, 5 show the diagram of structural model bootstrapping output without and with moderation, respectively. The validation of the proposed hypotheses can be examined using this model. A 95% confidence interval was taken for the bootstrapping and hypotheses validation.

**Figure 4:** Structural model bootstrapping without moderation. SC, Social Consciousness of Employees; Ent, Entertainment; Alt, Altruism; UVN, Unverified News Sharing; and CI, Corporate Image.

**Figure 5:** Structural model bootstrapping with Moderation. SC, Social Consciousness of Employees; Ent, Entertainment; Alt, Altruism; UVN, Unverified News Sharing; CI, Corporate Image; and WPS, Workplace Stress.

To examine whether the proposed hypotheses were accepted or rejected, the t-statistics and *p* value were considered. A value greater than 1.96 for t-statistics shows the acceptance of the hypothesis (Winship and Zhuo, 2020), while a value less than 0.05 for p value indicates that the hypothesis is accepted (Ioannidis, 2018). Besides this, the value of f^2^ or the effect size shows the impact of the independent variables (SC, Ent, Alt, and CI) on the dependent variable (UVN; Funder, 2019). The value of effect size (f^2^) near 0 shows the model strength is weak, while the value near 1 indicates a muscular model strength.

Table 4 shows the direct effects of the variables (direct effect of the independent variable on the dependent variable). H1 proposed that the SC of employee’s harm UVN. H1 got rejected as the results confirmed that (*O* = −0.052, *p* = 0.371, *t* = 0.895). F^2^ 0.003 shows a fragile model strength. H2 proposed that Ent impacts UVN. The results confirm the significant direct relationship between Ent and UVN with O 0.233, t-statistics 4.569, and value of *p* = 0.000. Thus, H2 got accepted. F^2^ 0.078 shows a weak model strength. H3 proposed that Alt impacts UVN. H3 got accepted as the results confirmed (*O* = 0.196, *p* = 0.001, *t* = 3.313). F^2^ 0.053 shows a weak model strength. H4 proposed CI harms UVN. The results showed a significant positive relationship between CI and UVN with O 0.513, t-statistics 8.097, and value of *p* = 0.000. Thus, H4 got rejected. F^2^ 0.211 shows a weak model strength.

**Table 4:** Direct effects of the variable.

**Paths**	**H**	**O**	**M**	**SD**	**t-statistics**	**Effect size (f** ^**2**^ **)**	**P value**	**Results**
**SC**➔**UVN**	H_1_	-0.052	−0.053	0.058	0.895	0.003	0.371	**Rejected**
**Ent**➔**UVN**	H_2_	0.233	0.234	0.051	4.569	0.078	0.000	**Accepted**
**Alt**➔**UVN**	H_3_	0.196	0.195	0.059	3.313	0.053	0.001	**Accepted**
**CI**➔**UVN**	H_4_	0.513	0.514	0.063	8.097	0.211	0.000	**Rejected**

*H, Hypothesis; O, Original Sample; M, Sample Mean, SD, Standard Deviation, SRMR = 0.075, NFI = 0.816, SC, Social Consciousness of Employees, Ent, Entertainment, Alt, Altruism, UVN, Unverified News Sharing, and CI, Corporate Image.*

Table 5 shows the indirect effects of the variable, i.e., in the mediator’s presence (CI). H5 proposed CI mediates the relationship between the SC of employees and UVN. The results confirm CI mediated the relationship between SC and UVN with O 0.328, t-statistics 7.080, and value of *p*. Thus, H5 got accepted. H6 proposed CI mediates the relationship between Ent and UVN. The results confirm CI mediated the relationship between Ent and UVN with O 0.093, t-statistics 4.010, and value of *p* = 0.000. Thus, H6 got accepted. H7 proposed CI mediates the relationship between Alt and UVN. The results confirm CI mediated the relationship between Alt and UVN with O 0.077, t-statistics 2.937, and value of *p* 0.003. Thus, H7 got accepted. F-square is the measure of standardized effect size. It shows the proportion of variance explained by the particular variable concerning the rest of the remaining variables. Effect sizes are usually larger if the variable under study shows higher variance than the rest of the independent variables or the total variance is higher. However, Funder (2019) have introduced new guidelines assuming that even an effect size of 0.05 shows a minimal effect size for this particular study, but this might have potential consequential and essential effects in the short run. Therefore, this study has reported even the weak effect sizes showing weak effect size but might be helpful in other contexts and helpful in future studies.

**Table 5:** Indirect effects of the variable.

**Paths**	**H**	**O**	**M**	**SD**	**t-statistics**	**P value**	**Results**
**SC**➔**CI**➔**UVN**	H_5_	0.328	0.326	0.046	7.080	0.000	**Accepted**
**Ent**➔**CI**➔**UVN**	H_6_	0.093	0.095	0.023	4.010	0.000	**Accepted**
**Al**➔**CI**➔**UVN**	H_7_	0.077	0.078	0.026	2.937	0.003	**Accepted**

*H, Hypothesis; O, Original Sample; M, Sample Mean; SD, Standard Deviation; SC, Social Consciousness of Employees; Ent, Entertainment; Alt, Altruism; UVN, Unverified News Sharing, and CI, Corporate Image.*

We conducted again the reliability and validity of the data with the moderator (i.e., WS) in the relationship between CI and UVN. The factor loadings, VIF, Cronbach Alpha, Composite Reliability, and AVE, were significant (see Table 6).

**Table 6:** Model assessment (moderation).

				**Construct reliability and validity**		
	**Factor loadings**		**VIF**	**Α**	**Composite reliability**	**AVE**
**Social Consciousness of Employees**	SC1	0.860	2.086			
	SC2	0.870	1.893	0.847	0.907	0.765
	SC3	0.894	2.239			
	Ent1	0.892	2.283			
**Entertainment**	Ent2	0.889	2.315	0.871	0.921	0.795
	Ent3	0.894	2.322			
	Alt1	0.910	4.239			
	Alt2	0.859	2.940			
**Altruism**	Alt3	0.890	3.858	0.925	0.943	0.736
	Alt4	0.910	4.034			
	Alt5	0.891	3.692			
	Alt6	0.759	1.510			
	UVN1	0.854	1.984			
**Unverified News Sharing**	UVN2	0.915	3.226	0.870	0.911	0.719
	UVN3	0.809	1.952			
	UVN4	0.808	2.110			
	CI1	0.738	1.339			
**Corporate Image**	CI2	0.854	1.696	0.736	0.850	0.655
	CI3	0.832	1.526			
	WPS1	0.864	4.554			
	WPS2	0.850	3.554			
**Workplace Stress**	WPS3	0.858	4.468	0.911	0.931	0.692
	WPS4	0.838	2.478			
	WPS5	0.812	2.643			
	WP6	0.763	2.148			

*SC, Social Consciousness of Employees; Ent, Entertainment, Alt, Altruism; UVN, Unverified News Sharing; CI, Corporate Image; WPS, Workplace Stress; VIF, Variance Inflation Factor; α, Cronbach Alpha, and AVE, Average Variance Extracted.*

Table 7 shows the moderating effect of the variable (i.e., WS). H8 proposed WS moderates the relationship between CI and UVN. The results confirm that WPS positively moderates the relationship between CI and UVN with t-statistics 2.278 and a value of *p* = 0.023 at a 0.05 level of significance. Thus, H8 got accepted.

**Table 7:** Moderating effects of the variable.

**Paths**	**H**	**O**	**M**	**SD**	**t-statistics**	**P value**	**Results**
**CI x WPS**➔**UVN**	H_8_	−0.077	−0.079	0.034	2.278	0.023	**Accepted**

*H*, *Hypothesis; O, Original Sample; M, Sample Mean; SD, Standard Deviation; UVN, Unverified News Sharing; CI, Corporate Image; and WPS, Workplace stress.*

## Discussion

This research focused on the determinants of UVN on SM and their impact on the CI in the current era. It was well established that these determinants positively or negatively influence the behaviors of the employees toward the news sharing on SM. It was also understood that the advent of technology to the next level creates enormous amounts of SM usage through different websites and platforms (Islam et al., 2020). It was also clear that SM was advancement in internetvtechnologies, and people started using SM for Ent, knowledge-seeking, and knowledge dissemination (Mustățea and Balaban, 2019). This research tried to differentiate between the social and environmental consciousness toward UVN. The results showed that SC alone does not affect UVN. It could be because social and environmental consciousness compels the business organizations’ users or employees to share practical information on SM. The concerned employees who are well conscious of their responsibilities tend to share only verified news instead of unverified or false news. Therefore, the hypothesis was rejected, unable to develop an association between the SC and UVN. Although it could direct the employees not to share such unverified news and could negatively affect it, it did not prove its worth in restricting unverified news.

Previously, many scholars looked into the relationships between social and environmental consciousness and intentions to share news and proved that, in specific contexts, such consciousness could influence news-sharing behaviors (Aldwairi and Alwahedi, 2018). They also stressed the importance of SC in the light of CSR practices which affluence the employees to share practical and reliable information on SM. Conversely, Ent and Alt developed an association with UVN, showing that the behavioral factors of Ent and Alt influence the sake of sharing news with the related people on SM. Many scholars have supported it in the recent past (Talwar et al., 2019). The scholars have previously affirmed that the Ent purpose of the employees motivates them to share every information they get, whether it is on the humorous side or the serious note. They only tend to share it without knowing the consequences (Balakrishnan et al., 2021). Even though some studies also found that shared news on SM, such as Twitter, revolved around the humorous aspect of disease spread, intended to reduce the anxiety among SM users during the recent pandemic (Chiodo et al., 2020). Similarly, Alt also pushed the employees to share the unverified news on the SM due to the underlying principle of Alt, which states that people tend to share the news and information with other people thinking of their benefit without getting back any benefit from them (Ma and Chan, 2014).

CI has been considered a beneficial aspect of organizational management while shaping a sustainable corporate resource. It worth has been proved many a time before as well. The CI leads to better organizational performance in a way that allows associated people get a view of it through its established image in the eyes of the stakeholders (Insch and Black, 2018). Therefore, it was assumed that CI could negatively disown the unverified news-sharing behavior of the employees on SM, but the results contradicted the assumption. The likely reason behind such results could be the impact of a CI on organizational performance. It could not shape the behaviors of the stakeholders involved with the organizations.

Although it was previously established that a full CI influenced the intention of sharing news about the organizations (Kim et al., 2020), that was only the intention of the stakeholders, not the behaviors. Moreover, the mediating role of CI in shaping the customers’ intention to buy from the firm proved its worth in the past, indicating that CI successfully aids in shaping the customer’s intentions toward the brand (Bataineh, 2015). This research also emphasized the information-sharing behavior of the people on SM sites. Our research also affirmed the mediating role of the CI between SC, Ent, Alt, and UVN. Such results lie because determinants of news sharing are not only the influencing factors for UVN. These are supported and carried out with the help of several other factors such as CI, which strongly mediated between these factors for the UVN behaviors. The negative association that could not be developed between SC and UVN was helped by the CI, because of the CI consciousness of the employees could minimize the sharing of unverified news and confined to sharing the verified news on SM only. Previously, no scholar investigated such relationships. WS strongly regulated the function of CI and UVN. This proved that uncontrolled WS plays a role in shaping employee’s negative behaviors. If given importance to reducing WS, it could shape the employees’ positive behaviors (Dimoff and Kelloway, 2019).

### Theoretical Implications

The theoretical implications are based on the findings got from the study. First, the empirical evidence strongly supports the relationship between Ent and UVN and Alt and UVN. These findings add to the existing literature on this topic. Second, the significant effect of the CI as a mediator provides convincing evidence that CI can facilitate the relationship between the SC of employees and UVN between Ent and UVN, and Alt and UVN. The study’s contribution in terms of these results enhances the reader’s knowledge of organizational dynamics. Last, the organizational behavior literature got enriched by the findings that WS moderates the relationship between CI and UVN.

### Practical Implications

The current study has few practical implications for managers and organizations. First, the role of corporate social responsibility (CSR) is crucial in filtering UVN and deteriorating the overall reputation of the organization. The corporate sector is quite vulnerable to UVN because various stakeholders are associated with this sector, thus CSR activities must be conducted from time to time. Moreover, the managers must consider the Ent of the employees to avoid the spread of UVN and deteriorating CI. Alt is another factor that fosters UVN and CI; therefore, altruistic values of the employees should be instigated to reduce the flow of UVN. Organizations must avoid controversial events that can be perceived as an unfavorable promotion by SM. A mechanism should be developed where the information is continuously monitored, including on social networking sites (SNSs). Organizations can decide the effect of negative information on SNSs. Furthermore, WS should be reduced in the organization. Organizations must develop favorable and supportive policies for the employees to keep CI and avoid UVN.

### Limitations and Directions for Future Research

The study’s limitations relate to the small sample size, which might affect data generalization. Thus, future studies can examine the results with a larger sample size. The study included employees of the corporate sector of China, which is the mainstream population in the post-Covid-19 situation when not everyone agrees to be part of the survey. Hence, future studies can include employees of other sectors as the telecommunication sector or FMCG working in other geographical regions. SC, Alt, and Ent have been used as the predicting variables for UVN; this model can be upgraded with other variables to get more insightful results about the factors that might affect the news sharing patterns. One factor can be the like and comment aptitude of the employees for no apparent reason to like the post. Future studies can use other mediating and moderating variables, such as corporate reputation, workplace safety and organizational environment.

## Conclusion

Organizations have switched their marketing and image building operations to SM to reach a maximum number of customers. Organizations run structure and campaigns to shape their CIs in this era of SM. In this whole scenario, the image building activities of the organization play a significant role. In this context, the SM teams even manipulate the facts by indulging in UVN. These deceptive and fake responses might affect the social standing of the organization and may tarnish the organization’s CI. Similarly, in this regard, CSR is crucial in reducing the effect of UVN on SM. The study examined the influence of SC on employees, Ent, and Alt on UVN with the mediation of CI and moderation of WS. The study concluded that the Ent and Alt of employees affect UVN. However, the direct negative effect of SC of employees and CI on UVN came out to be insignificant. The findings also showed that CI mediates the relationship between the SC of employees and UVN, Alt and UVN, and Ent and UVN. The moderating role of WS between CI and UVN was significant. It provides broader scope for organizations to protect their businesses through SM use and monitoring.

## Data Availability Statement

The original contributions presented in the study are included in the article/supplementary material; further inquiries can be directed to the corresponding authors.

## Ethics Statement

The studies involving human participants were reviewed and approved by Lanzhou City University, China. The patients/participants provided their written informed consent to participate in this study. The study was conducted in accordance with the Declaration of Helsinki.

## Author Contributions

ZZ conceived and designed the concept. SA collected the data. MA reviewed the paper. PC interpreted the data. All authors contributed to the article and approved the submitted version.

## Conflict of Interest

The authors declare that the research was conducted in the absence of any commercial or financial relationships that could be construed as a potential conflict of interest.

## Publisher’s Note

All claims expressed in this article are solely those of the authors and do not necessarily represent those of their affiliated organizations, or those of the publisher, the editors and the reviewers. Any product that may be evaluated in this article, or claim that may be made by its manufacturer, is not guaranteed or endorsed by the publisher.
